# miR-93, miR-373, and miR-17-5p Negatively Regulate the Expression of TBP2 in Lung Cancer

**DOI:** 10.3389/fonc.2020.00526

**Published:** 2020-04-28

**Authors:** Ye Li, Min Liang, Yunhui Zhang, Bing Yuan, Wenchao Gao, Zhizhou Shi, Jie Bai

**Affiliations:** ^1^Medical Faculty, Kunming University of Science and Technology, Kunming, China; ^2^First People's Hospital of Yunnan Province, Kunming, China

**Keywords:** lung cancer, TBP-2, miR-93, miR-373, miR-17-5p

## Abstract

Recently, several miRNAs have been revealed to play critical roles in oncogenesis and tumor progression of many cancers. Thioredoxin-1 (Trx-1) binding protein-2 (TBP-2) is an internal inhibitor of Trx-1, which plays the role in regulating oxidative stress, inhibiting cell growth, and promoting apoptosis. The expression of TBP-2 is usually decreased in cancer tissues. However, whether the miRNAs regulate the TBP-2 expression in lung cancer is still unclear. In this study, we examined the levels of TBP-2, miR-93, miR-373, and miR-17-5p in lung cancer tissues and their adjacent normal lung tissues of 36 patients. We found that the expressions of miR-93, miR-373, and miR-17-5p were higher, whereas the expression of TBP-2 mRNA and protein was significantly lower in lung cancer tissues compared with adjacent normal lung tissues. After the three miRNA mimics were transfected in the lung cancer cells, NCI-H460, the level of TBP-2 mRNA and TBP-2 protein was decreased. Then, the anti-cancer drug 5-fluorouracil was used to stimulate the NCI-H460 cells; the mRNA levels of miR-93, miR-373, and miR-17-5p were decreased, and the level of TBP-2 mRNA and protein was increased. Collectively, the above results suggest that miR-93, miR-373, and miR-17-5p negatively regulate the TBP-2 expression in lung cancer. This study may provide therapeutic targets with lung cancer.

## Introduction

Lung cancer is the most common malignant tumor in the world. The therapies for lung cancer have been improved much, such as surgical treatment, molecule-targeted therapy, and chemotherapy; however, the prognosis of patients with lung cancer is still unsatisfactory due to the high rate of metastasis and recurrence and the low rate of 5-years survival (1, 2). Therefore, developing novel therapeutic methods and understanding the mechanisms on lung cancer are very important.

MicroRNA (miRNA) is an important regulatory molecule involved in the tumorigenesis and development of cancer. It has been reported that miR-93, miR-373, and miR-17-5p were associated with hepatocellular carcinoma, breast cancer, gastric cancer, and lung cancer (3–6). Guan et al. reported that the expression of miR-93 was up-regulated and associated with lymph node metastasis stage in gastric cancer. The overexpression of miR-93 significantly enhanced the proliferation, migration, invasion, and epithelial–mesenchymal transition (EMT) of the gastric cancer (7). The miR-93 promoted gastric cancer metastasis by targeting interferon-alpha receptor-1 (IFNAR1) and activating the signal transducers and activators of transcription 3 (STAT3) signaling pathway (8). The high level of miR-93 was associated with poor patient survival, promoted lung cancer cell growth, and increased transforming growth factor (TGF)-beta-induced epithelial-to-mesenchymal transition via targeting disabled-2 (DAB2), zinc and ring finger 3 (ZNRF3), and neural precursor cell expressed developmentally down-regulated gene 4-like (NEDD4L) (9). The expression of miR-373 was decreased in non-small cell lung cancer (NSCLC), and overexpression of miR-373 suppressed cell EMT and the proliferation, migration, and invasion of NSCLC A549 cells by targeting beta-related factor 2 (BRF2) (10). The down-regulation of miR-373 enhanced lung cancer cells' radio-sensitivity and inhibited migration and invasion by targeting tissue inhibitor of metalloproteinases 2 (TIMP2) and regulating the phosphatidylinositol 3-kinase/protein kinase B (PI3K/AKT) and drosophila mothers against decapentaplegic protein (Smad) pathways (11). MiR-17-5p was overexpressed and correlated with the cell proliferation, invasion of carcinoma cells, and poor patient outcome (12). *Homo sapiens* HNF1A antisense RNA 1 long non-coding RNA (HNF1A-AS1) and lncRNA HNF1A-AS1 enhanced the proliferation and invasion of lung cancer cells by directly binding with and sponging miR-17-5p (13). Thus, miR-93, miR-373, and miR-17-5p might be the potential regulators of lung cancer. Although the prediction of miRNA targets database, TargetScan could predict some downstream of miR-373, miR-17-5p, and miR-93, such as Thioredoxin-1 (Trx-1) binding protein-2 (TBP-2). However, whether TBP-2 is the target of miR-93, miR-373, and miR-17-5p in lung cancer is still unknown.

In this study, we examined the levels of miR-93, miR-373, and miR-17-5p and the expression of TBP-2 in lung cancer tissues. We found that levels of miR-93, miR-373, and miR-17-5p were higher, whereas the expression of TBP-2 was lower in lung cancer tissues compared with adjacent normal tissues. We further found that miR-93, miR-373, and miR-17-5p could negatively regulate the expression of TBP-2 in NCI-H460 lung cancer cells.

## Methods

### Patients and Samples

Fresh lung cancer and adjacent normal tissues from 36 patients were collected. All the samples were residual specimens after diagnostic sampling. The primary tumor and the adjacent normal tissues from the same patient were separated and then immediately stored at −80°C. All lung cancer patients were hospitalized in the Department of Thoracic Surgery, the First People's Hospital of Yunnan province and treated with radical operation, and none of them received any preoperative treatments. All patients signed separate informed consent forms for sampling and molecular analysis. This study was approved by the Ethics Committee of the First People's Hospital of Yunnan Province, China.

### Cell Culture

NCI-H460 human lung cancer cells were cultured in Dulbecco's modified Eagle's medium (DMEM; Gibco, Grand Island, NY) with 10% fetal bovine serum (FBS), penicillin (100 U/ml), and streptomycin (100 mg/ml). All of these cells were maintained at 37°C in a humid atmosphere containing 5% CO_2_. 5-Fluorouracil (5-FU) was purchased from Sigma (St. Louis, MO, USA).

### Cell Transfection

The cells were seeded in six-well plates and transfected with miR-93, miR-373, and miR-17-5p mimics or mimic scramble negative control by using Lipofectamine 2000 transfection reagent (Invitrogen, Carlsbad, CA, USA) following the manufacturer's protocol. The mimics of miR-93, miR-373, and miR-17-5p and mimic scramble negative controls were synthesized by GenePharma (Shanghai, China).

### Total RNA Extraction and Real-Time PCR Assay

Total RNA was isolated from NCI-H460 cells by using TRIzol (CWBIO Corporation, Beijing, China) as described by the manufacturer and converted to cDNA using the RevertAid™ First Strand cDNA Synthesis Kit (Fermentas, Walldorf Baden, Germany).

Real-time PCR was performed to detect the relative level of TBP-2 expression. The PCR reactions were performed in a total volume of 25 μl, including 12.5 μl of Real-time PCR Master Mix, 1 μl of cDNA (5 ng/μl), and 1 μl of primer mix (10 μM each). PCR amplification and detection were performed by using the Prism 7300 Sequence Detection System (Applied Biosystems, Foster, CA, USA) as follows: an initial denaturation at 95°C for 2 min; 40 cycles of 95°C for 30 s, 59°C for 30 s, and 70°C for 1 min. The relative gene expression was calculated by using the comparative CT method. GAPDH was used as an internal standard for all samples. The sequences of primers are as follows: TBP-2 forward primer: 5′-GGATCCCAGCAGTGCAAAC-3′; TBP-2 reverse primer: 5′-AAGCCGAACTTGTACTCATATTTGT-3′; GAPDH forward primer: 5′-CAAGG CTGAGAACGGGAAG-3′; GAPDH reverse primer: 5′-GGTGAAGACGCCAGTGGACT-3′.

Hairpin-it^TM^ qRT-PCR Primer Set (GenePharma) was used for the measurement of the relative levels of miR-93, miR-373, and miR-17-5p. The mRNA expressions of miR-93, miR-373, and miR-17-5p were normalized to the expression of U6.

### Western Blot Analysis

Cells were detached with trypsin, centrifuged, and washed twice with pre-chilled phosphate buffer saline (PBS). Cell lysis buffer was subsequently added and incubated on ice for protein extraction. Protein concentration was determined by using the BCA Protein Assay Kit (Beyotime Biotechnology, China). Equal amounts of proteins were separated via 12% sodium dodecyl sulfate polyacrylamide gel electrophoresis (SDS-PAGE) and then transferred to a polyvinylidene fluoride (PVDF) membrane (Millipore Corporation, Billerica, MA, USA). The membrane was soaked in 10% skimmed milk (in PBS, pH 7.2, containing 0.1% Tween-20) for 2 h and incubated with an appropriate amount of primary antibody at 4°C overnight (anti-TBP2, 1:1,000, MBL international, Woburn, MA, USA; anti-β-actin, 1:5,000, Santa Cruz Biotechnology, CA, USA). Detection was performed by peroxidase-conjugated secondary antibodies (KPL, Gaithersburg, MD, USA) and chemiluminescence (Millipore Corporation, Billerica, MA, USA).

### Statistical Analysis

The data in this study are presented as mean ± standard deviation (SD) and statistically analyzed by using SPSS software (version 18.0, SPSS Inc., Chicago, USA). Two-tailed unpaired Student's *t* test was used to analyze the difference between two groups, normal non-cancerous tissues, and lung cancer tissues as indicated in corresponding figure legends. The one-way ANOVA followed by a Bonferroni's multiple comparisons test was used to compare the control and treated groups as indicated in corresponding figure legends.

## Results

### The mRNA Levels of miR-93, miR-373, and miR-17-5p in Lung Cancer and Adjacent Normal Non-cancerous Tissues

To investigate which miRNAs are involved in the development of lung cancer, we first detected the mRNA levels of miR-93, miR-373, and miR-17-5p in lung cancer and adjacent normal tissues of 36 samples by using Real-time qPCR. The mRNA levels of miR-93, miR-373, and miR-17-5p were higher in most carcinoma of the lung tissues compared with adjacent normal non-cancerous tissues. The folds of relative mRNA levels of miR-93, miR-373, and miR-17-5p in normal non-cancerous tissues and lung cancer tissues are shown in Figures 1A,C,E. The fold of cancer tissue to normal non-cancerous tissue in each sample was calculated by normal value as one. The level of miR-93 was higher in 26 of 36 lung cancer samples (72.2%) (*n* = 36, ^**^P < 0.01) (Figure 1B), miR-373 was higher in 28 of 36 lung cancer samples (77.8%) (*n* = 36, ^***^P < 0.001) (Figure 1D) and miR-17-5p was higher in 27 of 36 lung cancer samples (75%) (*n* = 36, ^**^P < 0.01) (Figure 1F), which suggest that higher expressions of miR-93, miR-373, and miR-17-5p are related to the lung cancer.

**Figure 1:** The mRNA levels of miR-93, miR-373, and miR-17-5p in lung cancer tissues. **(A,B)** The mRNA level of miR-93 in lung cancer tissues and adjacent non-cancerous tissues of 36 patients (*n* = 36, **P < 0.01, two-tailed unpaired Student's *t* test). **(C,D)** The mRNA level of miR-373 in lung cancer tissues and adjacent noncancerous tissues of 36 patients (*n* = 36, ***P < 0.001, two-tailed unpaired Student's *t* test). **(E,F)** The mRNA level of miR-17-5p in lung cancer tissues and adjacent noncancerous tissues of 36 patients (*n* = 36, **P < 0.01, two-tailed unpaired Student's *t* test).

### TBP-2 Expression in Lung Cancer and Adjacent Tissue

To investigate TBP-2 expression in lung cancer, we further detected the level of mRNA and protein of TBP-2 in lung cancer tissues and their compared normal non-cancerous lung tissues of 36 lung cancer samples by using Real-time qPCR and Western blot. The folds of relative mRNA level of TBP-2 in normal non-cancerous tissues and lung cancer tissues as shown in Figure 2A. The fold of cancer tissue to normal non-cancerous tissue in each sample was calculated by normal value as one. TBP-2 mRNA level was significantly lower in lung cancer tissues compared with non-cancerous tissues, 27 of 36 samples, which was 75% (*n* = 36, ^**^P < 0.01) (Figure 2B). The blots and folds of TBP-2 protein expression in normal non-cancerous tissues and lung cancer tissues are shown in Figures 2C,D. The fold of cancer tissue to normal non-cancerous tissue in each sample was calculated by normal value as one. The level of TBP-2 protein was remarkably lower in lung cancer tissues compared with the normal non-cancerous tissues, 30 of 36 samples, which was 83.3% (*n* = 36, ^***^P < 0.001) (Figure 2E). Contrary to the expressions of miR-93, miR-373, and miR-17-5p, the expression of TBP-2 was lower in lung cancer tissues.

**Figure 2:** The TBP-2 mRNA and protein levels in lung cancer tissues. **(A,B)** TBP-2 mRNA level in lung cancer tissues and adjacent non-cancerous tissues of 36 patients (**P < 0.01, two-tailed unpaired Student's *t* test). **(C–E)** TBP-2 protein expression in lung cancer tissues and adjacent noncancerous tissues of 36 patients (***P < 0.001, two-tailed unpaired Student's *t* test).

To compare the correlation between the mRNA levels of miR-93, miR-373, and miR-17-5p and the level of TBP-2 mRNA and protein, we organized change trends of the above results in Table 1.

**Table 1:** The change trends of levels of miR-93, miR-373, and miR-17−5p and the level of TBP-2 protein in lung cancer tissues compared to normal noncancerous tissues (36 samples).

**Patient#**	**TBP-2 prot (can vs. nor)**	**miR-93 (can vs. nor)**	**miR-373 (can vs. nor)**	**miR-17-5p (can vs. nor)**
1	Lower	Higher	Higher	Higher
2	Lower	Lower	Lower	Higher
3	Lower	Higher	Lower	Higher
4	Lower	Lower	Higher	Higher
5	Lower	Higher	Higher	Lower
6	Lower	Higher	Higher	Higher
7	Lower	Higher	Higher	Higher
8	Lower	Higher	Higher	Higher
9	Lower	Higher	Higher	Higher
10	Higher	Higher	Lower	Lower
11	Lower	Higher	Higher	Higher
12	Lower	Lower	Higher	Lower
13	Lower	Higher	Higher	Higher
14	Higher	Higher	Higher	Higher
15	Lower	Higher	Higher	Higher
16	Lower	Lower	Higher	Higher
17	Lower	Lower	Higher	Higher
18	Lower	Higher	Higher	Lower
19	Lower	Higher	Higher	Lower
20	Higher	Higher	Lower	Lower
21	Lower	Higher	Lower	Higher
22	Lower	Higher	Higher	Lower
23	Lower	Higher	Higher	Higher
24	Lower	Lower	Higher	Higher
25	Higher	Lower	Higher	Higher
26	Lower	Lower	Higher	Higher
27	Lower	Lower	Lower	Higher
28	Lower	Higher	Higher	Higher
29	Lower	Higher	Higher	Higher
30	Lower	Higher	Lower	Lower
31	Lower	Higher	Higher	Higher
32	Lower	Higher	Higher	Higher
33	Higher	Higher	Lower	Higher
34	Higher	Higher	Higher	Lower
35	Lower	Lower	Higher	Higher
36	Lower	Higher	Higher	Higher

*Text in red shows that the correlation between TBP2 and miRs is not always direct*.

### The Mimics of miR-93, miR-373, and miR-17-5p Reduced TBP-2 Expression in NCI-H460 Cells

To explore whether miR-93, miR-373, and miR-17-5p regulate the expression of TBP-2 in lung cancer cells, we transfected miRNA mimics into NCI-H460 cells and analyzed the expression of TBP-2. As shown in Figures 3A,B, the level of TBP-2 mRNA and protein was repressed after transfections of miR-93, miR-373, and miR-17-5p mimics, which suggest that the expression of TBP-2 is negatively regulated by miR-93, miR-373, and miR-17-5p in NCI-H460 cells (^**^P < 0.01) (Figures 3A,B).

**Figure 3:** MiR-93, miR-373, and miR-17-5p mimics inhibited the expression of TBP-2 in NCI-H460 cells. **(A)** The expression mRNA level of TBP-2 in NCI-H460 cells transfected by miR-93, miR-373, and miR-17-5p mimics (**P < 0.01, Bonferroni's multiple comparisons test). **(B)** The protein level of TBP-2 in NCI-H460 cells transfected by miR-93, miR-373, and miR-17-5p mimics (**P < 0.01, Bonferroni's multiple comparisons test).

### 5-FU Repressed the mRNA Levels of miR-93, miR-373, and miR-17-5p in NCI-H460 Cells

To explore whether miR-93, miR-373, and miR-17-5p are regulated by 5-FU in lung cancer cells, NCI-H460 cells were treated with 5-FU, 10 μM and 100 μM for 24 h, and the mRNA levels of miR-93, miR-373, and miR-17-5 were detected. The mRNA level of miR-93 was lower in 10 μM 5-FU-treated cells than control group cells (^*^P < 0.05) (Figure 4A), but there was no significant difference between 100 μM 5-FU-treated cells and control group cells. The mRNA level of miR-373 was lower in 5-FU-treated cells than control group cells (10 μM, ^*^P < 0.05, 100 μM, ^***^P < 0.001) (Figure 4B). The mRNA level of miR-17-5p was lower in 5-FU-treated cells than control group cells (10 μM, ^*^P < 0.05, 100 μM, ^**^P < 0.01) (Figure 4C). These data suggest that miR-93, miR-373, and miR-17-5p are involved in the oncotherapy of 5-FU in lung cancer cells.

**Figure 4:** 5-FU repressed the levels of miR-93, miR-373, and miR-17-5p in NCI-H460 cells. **(A)** The mRNA level of miR-93 was lower in 10 μM 5-FU-treated cells than control group cells (*P < 0.05, Bonferroni's multiple comparisons test) but not in 100 μM. **(B)** The mRNA level of miR-373 was lower in 5-FU-treated cells than control group cells (10 μM, *P < 0.05, 100 μM, ***P < 0.001, Bonferroni's multiple comparisons test). **(C)** The mRNA level of miR-17-5p was lower in 5-FU-treated cells than control group cells (10 μM, *P < 0.05, 100 μM, **P < 0.01, Bonferroni's multiple comparisons test).

### 5-FU Induced the Expression of TBP-2 in NCI-H460 Cells

We further examined whether 5-FU induces the expression of TBP-2 in lung cancer cells. We treated NCI-H460 cells with 10 μM and 100 μM 5-FU for 24 h and detected the expression of TBP-2. The mRNA level of TBP-2 was induced by 5-FU (10 μM, ^***^P < 0.001, 100 μM, ^**^P < 0.01) (Figure 5A), and the protein expression of TBP-2 was also induced by 5-FU (10 μM, 100 μM, ^*^P < 0.05) (Figure 5B), which suggests that TBP-2 is also involved in the oncotherapy of 5-FU in lung cancer cells.

**Figure 5:** 5-FU induced the expression of TBP-2 in NCI-H460 cells. **(A)** The mRNA level of TBP-2 was higher in 5-FU-treated cells than control group cells (10 μM, ***P < 0.001, 100 μM, **P < 0.01, Bonferroni's multiple comparisons test). **(B)** The protein level of TBP-2 was higher in 5-FU-treated cells than control group cells (10 μM, *P < 0.05, 100 μM, *P < 0.05, Bonferroni's multiple comparisons test).

## Discussion

Increased levels of miR-93, miR-373, and miR-17-5p were found in various types of cancers including lung cancer. In NSCLC, miR-93 expression was significantly correlated with survival rate, and silencing miR-93 expression might inhibit cell proliferation, migration, and invasion of lung cancer cells by targeting gene of phosphate and tension homology deleted on chromosome ten (PTEN) and retinoblastoma 1 (RB1) (14). It has been reported that miR-93 activated the PI3K/AKT signaling pathway and promoted tumorigenesis and metastasis of NSCLC via targeting liver kinase B1 (LKB1) (15). Qu et al. reported that miR-93 could down-regulate NEDD4L and increase TGF-induced EMT in lung cancer (9). MiR-93 regulates translocation of liposarcoma 1 (TLS1, FUS1), transducin repeat containing 2 (TRCP2), and disabled homolog 2 (DAB2), and plays an oncogenic role in lung cancer carcinogenesis. Gao et al. reported that miR-373 expression was decreased in glioma tissue specimens and cell lines and was involved in growth of cancer cells (16).

Trx-1 is a redox-regulating protein and plays a role in promoting growth of cells and inhibiting apoptosis. It has been reported that Trx-1 is increased and TBP-2 is decreased in various cancers. TBP-2 is the inhibitor of Trx-1 and inhibits the activity of Trx-1 by binding to its catalytic active center (17). TGF-beta1 and 1,25-dihydorxyvitamin D3 block the cancer cell cycle to inhibit cancer cell growth by increasing TBP-2 expression (18). In pancreatic tumor cells, miR-224 could enhance the proliferation and migration via directly targeting TBP-2 and activating downstream hypoxia-inducible factor-1 (HIF-1) signaling pathway (19). Park et al. found that downregulation of TBP-2 promoted the tumor growth by reducing p27 expression *in vitro* and *in vivo* in breast cancer (20). Interestingly, the bromodomain-containing protein 4 (BRD4) inhibitor, JQ1, induced apoptosis in acute myeloid leukemia cells by reactivating TBP-2 (21). Combination of mammalian target of rapamycin (mTOR) and histone deacetylase (HDAC) inhibitors could kill the NF-kB mutant and kirsten rat sarcoma viral oncogene (KRAS) mutant NSCLC cells by regulating the TBP-2/Trx-1 signaling pathway (22). Tyrosine kinase inhibitors (TKIs) inhibit the PI3K/Akt pathway in NSCLC cells and increase TBP-2 expression (23). It has been reported that Insulin-like growth factor 1 (IGF1) negatively regulates the expression of TBP-2 (24). Thus, TPB-2 plays an important role in inhibiting the growth of cancer cells.

MiR-373 negatively regulated TBP-2 expression and increased the expressions of HIF-1α and twist family basic helix-loop-helix transcription factor (TWIST). The miR-373/TBP-2/HIF1α/TWIST signaling axis was related to a poor prognosis of patients with breast cancer (25). MiR-17-5p inhibited TBP-2 expression during the senescence process. In senescent fibroblasts, TBP-2 expression is regulated by forkhead box O3 (FOXO3) and miR-17-5p (26). In the present study, we found that miR-93, miR-373, and miR-17-5p were higher and TBP-2 was lower in lung cancer tissues (Figures 1, 2). However, our results showed that the correlation between miRs and TBP-2 was not always direct in lung cancer tissues (Table 1). There are several possibilities: miR-93, miR-373, or miR-17-5p could, on their own, suppress the expression of TBP-2. The mechanisms on miRs regulate the expression of TBP-2 via different or complexed pathways. The reasons of the lung cancers are different. We further demonstrated that miR-93, miR-373, and miR-17-5p negatively regulated the expression of TBP-2 in NCI-H460 cells (Figure 3). To our knowledge, our results firstly revealed that miR-93 negatively regulated TBP-2 expression in lung cancer tissues and cells.

Ren et al. reported that miR-17-5p was up-regulated in HCT116/5-FU and SW480/5-FU cells. Silencing of miR-17-5p showed a suppressive role on cell viability, invasion, migration, and multi-drug resistance in HCT116/5-FU and SW480/5-FU cells (27). Xu et al. reported that hsa-miR-93 was involved in the cell proliferation and chemoresistance induced by 5-FU in HCC cells (28). TBP-2 was induced by 5-FU in colon carcinoma SW620 (29). We also investigated the correlation between miRs and TBP-2 after 5-FU treatment in NCI-H460 cells. Our results showed that the levels of miR-93, miR-373, and miR-17-5p were repressed and the expression of TBP-2 was induced by 5-FU (Figures 4, 5). Thus, 5-FU may induce the apoptosis in lung cancer cells by silencing miR-93, miR-373, and miR-17-5p and inducing TBP-2 expression.

In summary, our study showed that levels of miR-93, miR-373, and miR-17-5p were higher and the TBP-2 expression was lower in lung cancer tissues. MiR-93, miR-373, and miR-17-5p were inhibited and the expression of TBP-2 was induced by 5-FU. Thus, miR-93, miR-373, and miR-17-5p/TBP-2 pathways may be targets for lung cancer therapy.

## Data Availability Statement

The datasets generated for this study are available on request to the corresponding author.

## Ethics Statement

The studies involving human participants were reviewed and approved by Ethics Committee of First People's Hospital of Yunnan Province, China. The patients/participants provided their written informed consent to participate in this study.

## Author Contributions

JB and ZS conceived the idea and planned the study, wrote and reviewed the main manuscript. YL produced the figures and did statistical analysis. ML performed PCR and Western blot experiments. BY and YZ collected the samples of patients. WG performed cell experiments. All authors reviewed the manuscript.

## Conflict of Interest

The authors declare that the research was conducted in the absence of any commercial or financial relationships that could be construed as a potential conflict of interest.
